# Segmentation of Optic Disc and Cup Using Modified Recurrent Neural Network

This article has been retracted.

**DOI:** 10.1155/2022/6799184

**Published:** 2022-05-02

**Authors:** J. Surendiran, S. Theetchenya, P. M. Benson Mansingh, G. Sekar, M. Dhipa, N. Yuvaraj, V. J. Arulkarthick, C. Suresh, Arram Sriram, K. Srihari, Assefa Alene

**Affiliations:** ^1^Department of Electronics and Communication Engineering, HKBK College of Engineering, India; ^2^Department of Computer Science and Engineering, Sona College of Technology, India; ^3^Department of Electronics and Communication Engineering, Sri Ramakrishna Institute of Technology, India; ^4^Department of Electronics and Communication Engineering, Erode Sengunthar Engineering College, India; ^5^Research and Development, ICT Academy, IIT Madras Research Park, India; ^6^Department of Electronics and Communication Engineering, Karpagam Institute Technology, Coimbatore 641105, India; ^7^Department of Computer Science Engineering, Sri Ranganathar Institute of Engineering and Technology, Coimbatore, India; ^8^Department of Information Technology, AnuragUniversity, Hyderabad, India; ^9^Department of Computer Science and Engineering, SNS College of Technology, India; ^10^Department of Chemical Engineering, College of Biological and Chemical Engineering, Addis Ababa Science and Technology University, Ethiopia

## Abstract

Glaucoma is one of the leading factors of vision loss, where the people tends to lose their vision quickly. The examination of cup-to-disc ratio is considered essential in diagnosing glaucoma. It is hence regarded that the segmentation of optic disc and cup is useful in finding the ratio. In this paper, we develop an extraction and segmentation of optic disc and cup from an input eye image using modified recurrent neural networks (mRNN). The mRNN use the combination of recurrent neural network (RNN) with fully convolutional network (FCN) that exploits the intra- and interslice contexts. The FCN extracts the contents from an input image by constructing a feature map for the intra- and interslice contexts. This is carried out to extract the relevant information, where RNN concentrates more on interslice context. The simulation is conducted to test the efficacy of the model that integrates the contextual information for optimal segmentation of optical cup and disc. The results of simulation show that the proposed method mRNN is efficient in improving the rate of segmentation than the other deep learning models like Drive, STARE, MESSIDOR, ORIGA, and DIARETDB.

## 1. Introduction

Glaucoma is a long-term eye condition in which the optic nerve is gradually weakened due to increased pressure within the eye. A condition known as glaucoma affects around 60 million people globally and is the second biggest cause of blindness after cataracts. Glaucoma will affect an estimated 80 million individuals worldwide by 2020, according to current estimates [1]. Glaucoma can permanently damage the visual nerve if it is not detected early enough. Early detection of glaucoma is critical to ensuring that patients receive effective first-line medical treatment [2–4].

Finding the cup-to-disc ratio is a difficult, time-consuming, and expensive job that currently done solely by experts. Because of this, automated methods of glaucoma image detection and assessment are critical. To automatically detect the optic nerve head image, there are two methods [5]. Using image feature extraction for binary categorization of normal and abnormal circumstances is the first strategy. While clinical indications like the cup-to-disc ratio and inferior, superior, nasal, and temporal (ISNT) zones control the optic disc area in the second approach, it is less prevalent.

More than a million axons exit the retina and exit the eye through the scleral canal to carry visual information to the brain, all of which are contained in one little disc called the optic disc. In glaucoma, looking at the optic disc clarifies the link between optic nerve cupping and visual field loss [6]. Disc-to-cup ratio (DCR) is a measurement that compares the disc vertical diameter to the cup vertical diameter. Different techniques have been used for optic disc (OD), optic cup (OC) (Figure 1), or optic disc with optic cup segmentation.

In this paper, we develop an extraction and segmentation of optic disc and cup from an input eye image using modified recurrent neural networks (mRNN). The mRNN use the combination of recurrent neural network (RNN) with fully convolutional network (FCN) that exploits the intra- and interslice contexts.

The major contributions of the work involve the following:

- In preprocessing, we eliminate the duplication, similar data, null set, etc., and rest of other datas will be forward to next stage
- The proposed method FCN extracts the contents from an input image by constructing a feature map for the intra- and interslice contexts. This is carried out to extract the relevant information, where RNN concentrates more on interslice context
- The simulation is conducted to test the efficacy of the model that integrates the contextual information for optimal segmentation of optical cup and disc

## 2. Related Works

Using the Hough transform, Zhu and Rangayyan [7] devised an automatic segmentation approach for detecting the centre and radius of a circle that is close to the OD edge. This method was also utilised by Gonzalez and Woods [8] to find the OD edge. After normalising colour image components and converting them to luminance components, we thresholded the image effective region to figure out the reference intensity needed for circle selection.

For the OD automated segmentation, Welfer et al. [9] have developed a new adaptive technique that relies on anatomical models of vascular organisation combined with mathematical morphology. A two-stage methodology was used: first, the OD location was determined by analysing data from the main vessel arcade, where vessels were detected to determine the foreground and background images of the green channel. The background region was then identified by employing the RMIN operator, and the optic disc edge was then detected.

There is an algorithm proposed by Aquino et al. [10] that uses the localization methods to obtain an optic disc-like pixel from the OD. It utilises three distinct detecting strategies. For each approach, there is a candidate OD pixel, and a voting system is used to determine which pixel is the final classified one. The green channel was chosen because of its high level of contrast.

As an initial level set for the active contours used in optic disc segmentation, Tjandrasa et al. [11] utilised the Hough transform [12]. Prior to doing the image enhancement for OD segmentation, the image is converted to grayscale. In the next stage, the blood vessels are surgically removed to make the segmentation process go more smoothly. When low pixel values are detected, a threshold is used to blur the blood vessels. The median filter is then applied to soften the edges. A Hough transform is used to find a circle that matches the OD position in the image.

It was recently hypothesised that an edge detection method with a circular Hough transform and a statistically deformable model may be used to measure OD. The disc shape was modelled with the point distribution model using a number of landmarks. The image was analysed and the influence of blood vessels was reduced using a preprocessing procedure. Using a heuristic voting mechanism, the best channel was also found.

OD segmentation based on peripapillary atrophy removal was proposed by Cheng et al. [12]. There were three components to the algorithm: edge filtering, constraint elliptical Hough transformation, and the final step. Starting with a region of interest and then looking for the outer boundaries of that zone, this algorithm was built from there. The noise was removed using a low pass filter, and the first derivative from each row of the ROI was then calculated as described above. The detected disc boundary was used to determine a ring region, which was then divided into four equal sections to avoid spurious segmentation between the PPA and the OD.

According to Zhang et al. [13], a new OD localization method based on 1D projection has been developed. The horizontal position of OD was found using the vascular scatter degree. The brightness and edge gradients around OD were used to determine its vertical placement. Using a binary mask created by a morphological erosion technique, the retinal image region of interest could be located without resorting to further postprocessing. As a result of the preprocessing steps, a vertical window was created and moved over the vessels map to determine the degree of arterial scatter and find the OD horizontal placement using a 1D horizontal projection signal.

According to Fraga et al. [14], an approach for OD segmentation was developed that included many phases. The retinal image was normalised using the retinex algorithm to reduce contrast variability and improve process dependability. Both vessel convergence analysis and the fuzzy Hough transform are employed to find the optic disc location. The optical disc was found using both methods.

## 3. Joint OD Segmentation

The optic disc is a critical component of the retinal fundus image (RFI) [15] as in Figure 2. The study includes OD detection as a preprocessing component and then segmentation, which is a common step in most retinopathy screening procedures.

RNN stands for recurrent neural network, which is a deep representation of a neural network. It learns from the input sequence through nonlinear mapping and then transforms to a hidden state sequence to get the output. In RNN, the recurrent operation is accomplished by the use of an LSTM or recurrent unit. Using a recursive approach, hidden states are discovered by iterating over a recurrent module, which keeps the data in memory for a longer period of time. The process of obtaining important information from the provided input image makes it effective. After that, the recurrent unit is trained in the hidden states with LSTM to get the desired output.

Both LSTM and a linear fully connected layer are found in an RNN. The RNN extracts the ROI points from a normal eye image using the ROI points as an input. As a result, the RNN receives numerous images containing ROI points as input. On the input test image, the output obtains similar ROI points, where the ROIs are mapped based on ground truth data. The ROI feature vector has 1024 components, while the RNN generates 512 items as an output. The ROI vector on an input test image is output by the LFCL layer on LSTM cells placed on top of it.

Images having ROI patterns on the eyes are fed into the RNN to train it. Pupil, iris, and eyelid information are used to generate random ROI sites at the beginning of the process. After that, the patterns are repositioned to their original locations using ground truth values that provide enough background information. In the end, the ROI points are placed at the correction positions, i.e., on the upper and lower eyelids, corners, and the iris, after a number of iterations have taken place. The RNN's stability is critical because it causes the hidden layers to freeze, allowing the ROI points to be modified first and then the points in the neighbourhood. Training losses can be calculated by comparing the rebuilt ROI to the original ROI. This is calculated by adding up all of the squared errors in the eye region across all of the images.

(1) $$\begin{array}{c} E=\overset{N}{\underset{i=1}{\sum }}\left(\lambda_{e}{\left\|U\cdot \left(\beta \left(i\right)-\alpha \left(i\right)\right)\right\|}_{2}^{2}\right), \end{array}$$

where *N* is the eye images, *U* finds the shape of eye, *β* is the parameter vectors (estimated), *α* is the ground truth vector, and *λ* is the factor that helps in controlling the reconstruction of subset pairs.

The process flow of the proposed mRNN is given below.

After the detection of the optic disc, the optical cup is segmented using the segmentation process, which is given in the following section.

## 4. OC Segmentation Process

A section of the OD that is white and cup-shaped is the OC region. The optic disc connects the optic nerve to the retina at the back of the eye interior, in a circular area. From the retina in the eye, the optic nerve transmits sight-related impulses to the brain via the optic nerve. The optic disc at the back of the eye contains millions of retinal nerve fibres that bundle and travel to the brain through the optic nerve. When compared to the complete optic disc, the cup at the centre of the disc is fairly small.

An algorithm for segmenting the OC region (Figure 3) from the test image maps all ROI points or subset points. Iteration 2 of the algorithm includes instructions for separating out the regions of the eyes for segmentation. To exclude all noncontributing regions, we employ a background subtraction technique.

### 4.1. Sørensen-Dice Coefficients

Using a Dice coefficient, you may determine how similar two test images are by comparing their subset pairings. The Hausdorff distance is used to compare the distances between the similar subset pairs in the left OD and right OD image subsets *A* and *B*.

OC is then segmented, when the maximum distance between pairs of subsets exceeds a threshold value. It is possible to calculate the threshold distance by comparing the distance between two identical ROI spots on two distinct healthy OC images used as a ground truth.

The Hausdorff distance method measures the distance between the initial eye subset pairings in real-world images. When measuring Hausdorff distance, this distance is used to find amblyopia in a particular test image. The Sørensen-Dice coefficient is computed between the ground truth (*A*) and segmented OC (*B*), which is given below:

(2) $$\begin{array}{c} \text{SDC}=2\frac{\left|A\cap B\right|}{C\left(\left|A\right|+\left|B\right|\right)}, \end{array}$$

where *C* is the mean of *B*.

With regard to binary values, *a*_*i*_ and *b*_*i*_ refer to the two different groups of image pixels. This can be written as follows:

(3) $$\begin{array}{c} \left|A\cap B\right|=\underset{i}{\sum }a_{i}b_{i},\\ \left|A\right|=\underset{i}{\sum }a_{i},\\ \left|B\right|=\underset{i}{\sum }b_{i}. \end{array}$$

The OD pairs of left eye *A* and right eye *B* is regarded as a positive one and it is then calculated as below:

(4) $$\begin{array}{c} C=\frac{\sum_{i}a_{i}b_{i}}{\sum_{i}a_{i}\mathrm{sign}\left(b_{i}\right)}. \end{array}$$

The sign (*x*) function is represented as below:

(5) $$\begin{array}{c} \mathrm{sign}\left(x\right)=\left\{\begin{array}{cc} 1, & \text{if }x>0,\\ 0, & \text{if }x=0,\\ -1, & \text{if }x<0. \end{array}\right. \end{array}$$

∑_*i*_*a*_*i*_sign(*b*_*i*_) ∈ 0, OC subset fails to overlap, and then *C* is assigned as unity upon *a*_*i*_ ∈ 0, 1. Here, the values are considered binary if *C* and ∑_*i*_*a*_*i*_*b*_*i*_ = 0.

## 5. Results and Discussions

In this section, we present the comparative results between the proposed method and existing methods in terms of various performance metrics including accuracy, F-measure, specificity, sensitivity, and mean average percentage error. The comparison is conducted in terms of various datasets that includes Drive [16], STARE [17], MESSIDOR [18], ORIGA [19], and DIARETDB0 [20]. The simulation is conducted on a high-end computing system running on a Ryzen 5 powered 4500 CPU with 16 GB RAM and 4 GB GPU. The results of training the segmentation algorithm are given in Figures 4 and 5, and the validation of segmentation is given in Figure 6.

Table 1 shows the training and testing time of segmenting the OC after the detection OD. The results show that the testing of classifier is effective since it offers a marginal difference with the testing results.

Figure 7 shows the results of proposed mRNN segmentation algorithm against various existing methods including level set method, FCM, and ANN. The results of simulation on various datasets show that the proposed method achieves higher rate of segmentation accuracy than other methods.

Figure 8 shows the results of sensitivity between the proposed mRNN segmentation algorithm against various existing methods including level set method, k-means, FCM, and ANN. The results of simulation on various datasets show that the proposed method achieves higher rate of sensitivity than other methods.

Figure 9 shows the results of specificity between the proposed mRNN segmentation algorithm against various existing methods including level set method, FCM, and ANN. The results of simulation on various datasets show that the proposed method achieves higher rate of specificity than other methods.

Figure 10 shows the results of F-measure between the proposed mRNN segmentation algorithm against various existing methods including level set method, FCM, and ANN. The results of simulation on various datasets show that the proposed method achieves higher rate of F-measure than other methods.

Figure 11 shows the results of F-measure between the proposed mRNN segmentation algorithm against various existing methods including level set method, FCM, and ANN. The results of simulation on various datasets show that the proposed method achieves higher rate of F-measure than other methods.

## 6. Conclusions

In this paper, we develop an extraction and segmentation of OD and OC from an input eye image using mRNN. The mRNN use the combination of RNN with FCN that exploits the intra- and interslice contexts. The FCN extracts the contents from an input image by constructing a feature map for the intra- and interslice contexts. This is carried out to extract the relevant information, where RNN concentrates more on interslice context. The simulation is conducted to test the efficacy of the model that integrates the contextual information for optimal segmentation of optical cup and disc. The results of simulation show that the proposed method is efficient in improving the rate of segmentation than the other deep learning models. In future, the proposed modelling can improvised with the several utilization of machine learning or deep learning methods.

## Figures and Tables

**Figure 1:** Retinal fundus image—OD and OC.

**Figure 2:** Flowchart for proposed algorithm.

**Figure 3:** OC region (the layer while in the centre of eye ball—white region).

**Figure 4:** The results of training the segmentation algorithm, where red denotes the proposed method, blue denotes the level set method, black denotes the FCM, and green denotes the ground truth.

**Figure 5:** After training the segmentation of OC is conducted with original images (a–c) and then on preprocessing (a1–c1), feature extraction (a2–c2), detection of OD (a3–c3), and segmentation of OC (a4–c4).

**Figure 6:** The results of testing the segmentation algorithm, where red denotes the proposed method, blue denotes the level set method, black denotes the FCM, and green denotes the ground truth.

**Figure 7:** Segmentation accuracy of OC with OD detection.

**Figure 8:** Sensitivity of OC with OD detection.

**Figure 9:** Specificity of OC with OD detection.

**Figure 10:** F-measure of OC with OD detection.

**Figure 11:** MAPE of OC with OD detection.

**Algorithm 1:** Detection of OD region.

**Algorithm 2:** Segmentation of OC.

**Table 1:** Training and testing time of segmenting the OC.

Images	Training	Testing
Image 1	9953 s	10121 s
Image 2	10251 s	11299 s
Image 3	12418 s	12658 s

## Data Availability

The datasets used and/or analysed during the current study are available from the corresponding author on reasonable request.
